The article "Advocacy for the Development of Teacher Leadership in the Context of ECC Reforms in China" was published in 2022. Journal: Comput Intell Neurosci.

# Advocacy for the Development of Teacher Leadership in the Context of ECC Reforms in China

**DOI:** 10.1155/2022/8204999

**Published:** 2022-07-14

**Authors:** Xiaoyan Shen

**Affiliations:** School of ECE, Shanghai Normal University Tianhua College, Shanghai, China

## Abstract

China's development is inseparable from the reform of education, so ECE is very important in the development of Chinese society. Based on this reason, this paper introduces the three reform waves of communist Chinese society under the influence of western culture. Because the professional level of kindergarten teachers does not match the concepts and requirements of the three preschool curriculum reforms in Chinese society, this paper analyzes the solutions based on this problem and holds that the leadership of kindergarten teachers should be vigorously developed.

## 1. Introduction

China has long recognized the important role of ECE in children's development [1]. Under the mutual influence of Chinese local culture and western culture, China's ECE has experienced many landmark changes. This paper introduces the changes of Chinese social culture under the influence of Chinese traditional local culture and western culture under communism. There have been three reforms of preschool education. For more than a century, China's educational practice has been influenced by Chinese traditional culture and Soviet thoughts, and it is also hoped to learn from advanced western educational ideas and methods and actively explore educational practices suitable for China. Although the third comprehensive reform of ECE has made great progress and had a wide impact on society, there are still many problems. One of the outstanding problems is that the quality of kindergarten teachers does not match the idea and demand of education reform. Some experts point out that teachers play an important role in the new curriculum reform. Focusing on the development of teachers' leadership is the most reliable solution under the mutual influence of Chinese native culture and western culture.

## 2. The Current Situation of ECE and Care in China

Preschool education refers to the education of children from 0 to 6 years of age. In recent years, the age range of children enrolled in kindergartens in some provinces has also begun to expand, meaning that children aged 2-3 can also enter the kindergarten [3].

In China's education system, ECE belongs to basic education, but not to nine-year compulsory education (six years of primary school and three years of middle school), which will get more education budget from the government. In all the stages of basic teaching, the budget for ECE is the least. For example, ECE has received only 1.3-1.4% of the national education budget in the last 17 years in China [4].

The article "Advocacy for the Development of Teacher Leadership in the Context of ECC Reforms in China" was published in 2022. Journal: Comput Intell Neurosci.

With the Third Plenary Session of the Eleventh Central Committee in 1978, China began to implement the policy of internal reform and opening to the outside world. Under the influence of the reform and opening-up policy, all walks of life in China have undergone earth-shaking changes, including preschool education, and the reform results of preschool education are the most remarkable [5]. As a result, there has been noticeable and dramatic improvements in ECE. However, there were still many challenges and difficulties to be solved by Chinese early education professionals [6]. One of the prominent issues was that the professional development level of most early childhood educators cannot meet the requirements of the reform. In response to this phenomenon, this paper attempted to propose the advocacy from the social and historical aspect of ECC reforms and the influence of the hybrid of three cultures on the reform.

## 3. A Social and Historical Aspect of ECC Reforms in China

In the past decades, under the interaction between Chinese local culture and foreign culture, especially western culture, a series of tremendous changes have taken place in ECE in China. In China, ECE is a full-time program of primary education for children. Generally speaking, the need to verify the quality of ECE starts with examining the characteristics of the curriculum, which is the key core of education [7].

In the development of ECE in China, the early childhood curriculum (ECC) reform mainly went through three stages, which were, respectively, affected by the social development and cultural characteristics at that time. The three stages of ECC reform, along with the historical process of major social changes of different origins, took place in 1920s to 1940s, 1950s to 1960s, and 1980s to the present, respectively [8].

### 3.1. The ECC Reform from 1920s to 1940s

The formal development of ECE in China began in the early 20th century. In 1903, China's first kindergarten was established in Wuhan (Zhu & Zhang, 2008), which copied the Japanese education model from the content and methods to the toys and facilities [9]. At that time, the influence of western missionaries was very extensive, and China's ECE also received its influence.

The May 4th New Culture Movement broke out in 1919, created conditions for the spread of various western educational thoughts in China, and had a profound influence on the reform of modern education in China, among which the ideological influence of John Dewey was particularly obvious [10]. In addition, the famous western scholars of ECE at that time, such as German Froebel and Italian Montessori, and their ECC models also became the object of imitation and learning for Chinese teachers [11].

The article "Advocacy for the Development of Teacher Leadership in the Context of ECC Reforms in China" was published in 2022. Journal: Comput Intell Neurosci.

However, local Chinese educators such as Chen Heqin, Tao Xingzhi, and Zhang Xuemen also had insight into the disadvantages brought about by copying foreign countries in ECE, which did not adapt to the social and cultural conditions in China at that time, and put forward the idea of starting with ECC reform to make ECC scientific and localized [12]. A curriculum called “unit integrated curriculum” was implemented in Nanjing in 1923, which initiated the first ECC reform (1920s–1940s) in China. In theory, it confirmed the subjectivity of children in the curriculum, and the curriculum should include all activities of children in kindergarten.

### 3.2. Full Acceptance of Soviet Theory (1950s–1960s)

After the founding of the People's Republic of China in 1949, under the background of comprehensive learning from the Soviet Union, ECC also fully accepted the theory and practical experience of the Soviet Union. In the 1950s, China began the second ECC reform. Although the Chinese ECC no longer used the word “curriculum,” it actually reflected a narrow understanding of the curriculum at that time, that is, the curriculum was regarded as a subject, and children were educated through the teaching of various subjects in kindergartens [13]. The Chinese Ministry of Education had completely rejected the previous practice, requiring kindergartens to systematically teach young children through “homework,” emphasizing the leading role of teachers, and attaching importance to the learning of knowledge and skills for young children.

From 1966 to 1976, the “Cultural Revolution” occurred in China, which made China's education suffer a catastrophe, and ECE was no exception. That period was known as the dark period of ECE in China [14].

### 3.3. Progress for the Third ECC Reform (1980s to the Present)

After the ten-year Cultural Revolution from 1966 to 1976, Chinese leader Deng Xiaoping put forward the famous reform and opening-up policy [15]. This reform has changed China's traditional education concept and made China's ECE go out of the dark period and turn into the golden period of ECE. After about 30 years of efforts, China's ECE reform has made great achievements [16].

Since the 1980s, Chinese early childhood educators have launched a large-scale ECC reform movement with ECC reform as a breakthrough point. Various foreign child development and education theories, such as Montessori, Dewey, Bronfenbrenner, Bruner, and especially Piaget's ideas, began to spread widely, and the thoughts of modern educators in China, especially those of Chen Heqin, were emphasized again, which provided theoretical background for the ECE reform since the 1980s [11]. Since then, the influence of the Soviet Educational theory on ECE in China has gradually weakened.

The article "Advocacy for the Development of Teacher Leadership in the Context of ECC Reforms in China" was published in 2022. Journal: Comput Intell Neurosci.

The third ECC reform started from the spontaneous experiment of China's kindergartens and played a great role in promoting it. In 1989, China's education authorities issued the Kindergarten Work Regulations (trial version). Since then, ECC reform has been transformed into a “top-down” reform led and promoted by the national administrative power [17]. In order to further deepen this reform, in 2001, the Ministry of Education issued the Supplementary Guidelines for Kindergarten Education Practice (trial version). These reforms and policies are aimed at the previously long-existing teacher-centered curriculum system, which has shifted to emphasizing the development of children and taking plays as basic activities [18]. The Supplementary Guidelines issued in 2001 reflected the core concept of ECC reform to provide integrated, situational, and life-oriented experience for children. Taking the five fields of “health, language, society, science, and art” as examples, the curriculum objectives, contents, and requirements as well as guiding points were elaborated [19].

Furthermore, during this reform period, some well-known western curriculum models such as Project Approach in the United States, Reggio Emilia Practice in Italy, and Montessori curriculum mode in Italy were widely known by Chinese ECE scholars and gradually localized in some kindergartens [20]. In addition, Chinese early education experts have also developed local curriculum based on China's national conditions and social needs, such as the theme-based integrated curriculum led by Zhu Jiaxiong [21], and the Anji Play Approach developed by Cheng Xueqin [22].

The reform in this stage is still going on, and its scale, length of time, and amount of resources are unmatched by previous ECC reforms. However, with the development of society and the passage of time, people began to evaluate this reform from multiple perspectives and put forward many problems at the conceptual and practical levels [23].

## 4. A Mixture of Three Cultures in China

China's ECC reform in these three stages happened to be accompanied by great social changes, and all of them were influenced by foreign cultures without exception. Unfortunately, the introduced curriculum did not necessarily meet the needs of Chinese children nor did ECE teachers in China have the expertise to handle it. This also reflects the need to pay enough attention to cultural compatibility in the ECC reform in China [24]. That is to say, the mixture of three cultures: Chinese native culture, Soviet Union (communist) culture, and western culture, has an indelible impact on China's social changes, including different aspects of ECC reform [25].

The article "Advocacy for the Development of Teacher Leadership in the Context of ECC Reforms in China" was published in 2022. Journal: Comput Intell Neurosci.

As is known to all, Chinese native culture originated from Confucianism, which had exerted a far-reaching and comprehensive influence on the Chinese people. The impact on education lied in the emphasis on repetition and memorization of individuals rather than encouraging and fostering creativity and flexibility. In the ECC reform, although Chinese teachers accepted the curriculum or pedagogies of foreign culture, they still adopted traditional teaching methods in practice because of the long-term influence of deep-rooted Confucianism [26].

The influence of Soviet culture is mainly reflected in China's second-stage ECC reform, which was generally stable and smooth. Traditional Chinese culture and communist culture were compatible to a certain extent because both value centralized management, planning systems, learning outcomes, clear goals, and teachers' guidance.

As a representative of western culture, the United States put forward a famous open door policy. Under the influence of this policy, the advantages of other cultures also had an impact on the third reform of China's preschool education. Although many ECE practitioners in China imitate the western education methods and try to change the traditional teaching methods from adult-centered to child-centered, they find that there are still many shortcomings to be improved in the process of teaching practice, and these problems cannot be solved in a short time [27].

The influence of these three cultures on ECE is not immutable, but developed dynamically, and each one had an impact on different aspects of ECC. Sometimes two cultures could produce a combined influence, for example, the commonality of Chinese native culture and communist culture strengthened the authority of teachers, and sometimes the influence of two cultures would offset each other to a certain extent, for instance, collectivism in Chinese native culture was the exact opposite of the cultivation of individuality in western culture.

## 5. One Noticeable Issue in ECC Reform: EC Teachers' Professional Level Did Not Match the Requirement

As mentioned above, EC teachers in China have been fully affected by the ECC reform. They have recognized the importance of learning child-centered educational theories and also have tried to change the traditional education system centered on knowledge transfer and skill acquisition, but it was still difficult to get rid of the old curriculum mode and traditional teaching methods in practice [28]. Early educators want to achieve results in the reform of ECE, so they can learn about the children's experiences, interests, and wants of the objects of education before teaching practice, which is very significant for the improvement of teaching effect [22]. With the advancement of the third phase of ECC reform, many methods and practices in the field of early education have been implemented, but few have achieved success, especially in developing regions of China. New cognition may not necessarily have an impact on traditional teaching methods.

The article "Advocacy for the Development of Teacher Leadership in the Context of ECC Reforms in China" was published in 2022. Journal: Comput Intell Neurosci.

In the exploration of preschool teaching reform, many preschool teachers are not clear about the main purpose of teaching, and the meaning of teaching is rather vague, especially in the complicated and changeable teaching environment at that time [29]. With the development of preschool education reform, preschool education requires higher and higher professional level of preschool teachers. However, the current problem is that the professional level of preschool teachers cannot meet the requirements of preschool education reform, which is the most important problem to be solved in preschool education reform and the key to the success of the reform.

The ultimate goal of the reform is to make both teachers' teaching and students' learning meaningful. As the first contact with children, teachers have the most say in the practicality and effectiveness of the curriculum. Therefore, in the development and implementation of a new curriculum, teachers should also have certain decision-making power, which requires them to achieve more professional levels [30]. The Chinese government is launching actions to promote EC teachers' professional development. One of its views is that EC teachers should participate in school-based research and reflect their own classroom behavior and be able to strike a certain balance between their preset learning tasks and activities of interest to children.

The main problems in the third reform of ECE in Chinese society are that the professional level of early childhood teachers cannot meet the requirements of the latest early childhood teaching level and the number of early childhood teachers is insufficient. To make the teaching reform successful, we must put forward concrete and effective solutions to these two problems. In order to solve these two main problems, the Chinese government has set up three levels of training programs for preschool teachers, namely, the national level, the provincial level, and the municipal level [31]. The kindergarten teachers who receive training have different teaching levels and regions, so different types of training programs should be set up according to different kindergarten teachers' needs. However, at present, most preschool teaching and training programs are not aware of this problem but blindly study the western preschool teacher training courses. As the training courses for preschool teachers are not targeted, the training effect for preschool teachers is not very satisfactory at present. Therefore, there is still a certain gap between the overall professional level of preschool teachers and the professional level required by preschool education reform. The third preschool education reform in China has not achieved obvious results [32].

The article "Advocacy for the Development of Teacher Leadership in the Context of ECC Reforms in China" was published in 2022. Journal: Comput Intell Neurosci.

## 6. Developing Teacher Leadership as a New Direction for the ECC Reform

At present, as the connection between countries in the world is increasing, if you want to gain an advantage in the competition in this era of globalization, you must make teaching develop with the times. So, countries all over the world have started their own educational reforms. Southeast Asian countries have borrowed the teaching mode of distributed leadership from the ECE reform in western developed countries. It can be seen that teacher leadership is very similar to distributed leadership, which is another form of distributed leadership.

Relevant scholars have found in the exploration of ECE reform that teacher leadership plays a crucial role in the quality of teaching and the success of teaching effect. Although teacher leadership is a decisive factor for the success of teaching, there is no unified explanation for the definition of teacher leadership in the field of early childhood teaching reform. The term “agent” means “a person or group responsible for leading change at the school level.” Relevant scholars involved in the reform of ECE think that teachers who are “agents” can be divided into two different leadership roles in performing administrative and teaching duties, namely, formal leadership role and informal leadership role. Teachers' role in schools has been expanded, and they participate in school-related affairs, including curriculum development, staff training, school improvement, personnel affairs, school management, and decision making, instead of being confined to classroom teaching.

Ho Tikly (2012) found that in the process of preschool education reform, preschool teachers who have been receiving professional training have realized their leading role in the education process. However, under the influence of this out-and-out educational reform and innovation and different cultures, at present, the professional level of most preschool teachers still cannot reach the level required by preschool education reform, so there is still a long way to go for the success of preschool education reform in China. This paper holds that promoting the development of teachers' leadership can make preschool teachers change from passive recipients to initiators of preschool education reform, which will achieve more effective results in solving the above problems.

The article "Advocacy for the Development of Teacher Leadership in the Context of ECC Reforms in China" was published in 2022. Journal: Comput Intell Neurosci.

## 7. Conclusion

Under the guidance of the reform and opening-up policy, the Chinese government has learned from the west, making various fields develop towards diversification. Through the combination of the three ECE reforms and the latest ECE reform and development goals proposed by the Chinese government, the development of preschool teachers' leadership can enable them to have more opportunities to participate in the decision making of teaching reform and thus have more active decision-making power, which has a very significant effect on mobilizing the enthusiasm of preschool teachers. This may be a feasible method for improving the professional level of teachers under the specific cultural soil and era background.

## Data Availability

The data used to support the findings of this study are available from the corresponding author upon request.
